The article "MiR-375-3p Promotes Cardiac Fibrosis by Regulating the Ferroptosis Mediated by GPX4" was retracted in 2023. Reasons: signs of a paper mill; compromised peer review; unreliable results or conclusions.

# MiR-375-3p Promotes Cardiac Fibrosis by Regulating the Ferroptosis Mediated by GPX4

**DOI:** 10.1155/2022/9629158

**Published:** 2022-04-22

**Authors:** Yu Zhuang, Dicheng Yang, Sheng Shi, Limin Wang, Min Yu, Xiangdong Meng, Yongliang Fan, Ren Zhou, Feng Wang

**Affiliations:** ^1^Department of Cardiovascular Surgery, Shanghai General Hospital, Shanghai Jiao Tong University School of Medicine, Shanghai 200080, China; ^2^Department of Cardiothoracic Surgery, Shanghai Ninth Hospital, Shanghai Jiao Tong University School of Medicine, Shanghai 200011, China

## Abstract

Although coronary artery recanalization after myocardial infarction improves patient outcomes, inadequate ventricular remodeling following ischemia-reperfusion (IR) injury and secondary cardiac fibrosis (CF) are common and can lead to heart failure. MicroRNAs (miRNAs) play an important role in cardiovascular disorders. However, the underlying molecular mechanism of miRNAs in the occurrence and progression of CF has not been fully elucidated. Herein, through the construction of an I/R rat model and an angiotensin II-induced CF cell model, we evaluated the role of miR-375-3p in the progression of CF. In the I/R rat model and CF cell model, miR-375-3p promoted fibrosis by accelerating the ferroptosis of cardiomyocytes through mediating glutathione peroxidase 4 (GPX4). Furthermore, we treated the rats or cell model with miR-375-3p antagomir (or inhibitor) and ferroptosis inhibitor Ferrostatin-1 (Fer-1). The results showed that miR-375-3p antagomir (or inhibitor) and Fer-1 promoted the antioxidant capacity of cardiac fibroblasts, reduced GPX4-mediated ferroptosis process and alleviated I/R-induced CF. In conclusion, this study revealed that miR-375-3p directly targeted GPX4—an inhibitor of the ferroptosis pathway. Meanwhile, miR-375-3p can be a new potential biomarker for the prevention and treatment of CF.

## 1. Introduction

Heart failure (HF), a multifactorial disorder that is usually the end stage of many cardiovascular diseases (CVD) [1], is a global pandemic with an increasing incidence [2]. Myocardial infarction (MI) is a common coronary artery disease and the main inducement of HF. Acute MI with vascular occlusion not only causes loss of myocardium, but also leads to ventricular remodeling and chronic HF [3, 4]. Early restoration of vascular perfusion can reduce myocardial necrosis and remodeling, and improve patient prognosis. After myocardial tissue reperfusion, the resulting myocardial damage and functional deterioration will induce myocardial cell necrosis, which is called ischemia-reperfusion (IR) injury [5, 6]. Cardiac fibrosis (CF) is also an important part of ventricular remodeling after MI and is closely related to HF. During this process, cardiac fibroblasts are activated to become myofibroblasts [7, 8]. Subsequently, type I and III collagen mediate the excessive deposition of extracellular matrix, accompanied by elevated expression of transforming growth factor *β*1 (TGF-*β*1) [9, 10]. However, currently, the molecular mechanisms regulating CF development remain to be elucidated.

The article "MiR-375-3p Promotes Cardiac Fibrosis by Regulating the Ferroptosis Mediated by GPX4" was retracted in 2023. Reasons: signs of a paper mill; compromised peer review; unreliable results or conclusions.

Ferroptosis is a novel type of programmed cell death characterized by an increase in iron-dependent reactive oxygen species (ROS) [11]. Ferroptosis is closely related to various pathological processes, and participates in the occurrence and development of many diseases such as tumors, IR injury and neuropathy [12–15]. The occurrence of ferroptosis involves a variety of pathways such as inhibition of glutamate-cystine transport, oxidative stress, abnormal iron metabolism and lipid peroxidation [16]. Glutathione peroxidase 4 (GPX4) is a cofactor of glutathione (GSH), which can effectively remove excessive ROS in cells. The activity of GPX4 is lost in the presence of ferroptosis, while the expression of COX2, ACSL4, PTGS2, and NOX1 was upregulated [17, 18]. Research has shown that ENPP2/LPA protected cardiomyocytes from ferroptosis by regulating the expression of GPX4 and enhancing Akt signaling [19]. Therefore, targeting ferroptosis may be a new approach to prevent and treat heart diseases such as IR and CF.

MicroRNAs (miRNAs) are noncoding RNAs (ncRNAs) consisting of only 18–25 nucleotides. By binding to target mRNAs, miRNAs inhibit the translation of mRNAs or promote their degradation to play a biological role. In addition, miRNAs play a key role in maintaining normal heart development and the pathogenesis of cardiovascular diseases such as IR and CF [20, 21]. For example, down-expression of miR-27a in CF cells reduced the expression of collagen and inhibited the fibrotic response [22]. In this study, the effect of miR-375-3p on CF was investigated by constructing a CF rat model, and whether miR-375-3p regulates GPX4-mediated ferroptosis in the progression of CF was explored. It was found that miR-375-3p directly targeted the mRNAs of ferroptosis regulator GPX4. In the rat model of CF, the expression of miR-375-3p was elevated along with increased ferroptosis signaling in cardiomyocytes. Our research reveals a new mechanism of CF after MI and provides miRNA-based intervention strategies.

## 2. Materials and Methods

### 2.1. Establishment of an IR Rat Model

Forty-two SD rats were randomly divided into sham operation group (*n* = 6) and I/R model group (*n* = 36). In the model group, rats were ligated with left anterior descending coronary artery to simulate MI. Specifically, after anesthetizing the animals in the I/R model group, an oblique incision was made in the third and fourth intercostal spaces of the left chest to expose the heart. Under a stereomicroscope, the junction of the pulmonary artery cone and the left atrial appendage was ligated with 6/0 noninvasive suture needle silk threads at 1-2 mm below the starting point of the coronary artery. Successful ischemia was indicated by ST segment elevation or *T* wave height and peaks of MI performance on electrocardiogram (ECG). The ligation was stopped after 45 minutes of ischemia, and the rats were maintained for 24 hours after reperfusion. As a drug treatment, 6 I/R model rats were treated with 20 nmol miRNA NC inhibitor (Thermo Fisher Scientific, Waltham, MA), 20 nmol miR-375-3p antagomir (Thermo Fisher Scientific, Waltham, MA) and 2 mg/kg Ferrostatin-1 (Fer-1; MCE, USA) for 28 days. The myocardial tissues of rats in the sham operation and I/R model groups as well as I/R model drug treatment group were then used for subsequent testing.

The article "MiR-375-3p Promotes Cardiac Fibrosis by Regulating the Ferroptosis Mediated by GPX4" was retracted in 2023. Reasons: signs of a paper mill; compromised peer review; unreliable results or conclusions.

### 2.2. Culture of Cardiac Fibroblasts

The heart tissue of newborn SD rats was cut into pieces after washing with precold PBS and 40 minutes of digestion with 2.0 g/L type II collagenase (Yeason, China) and 2.5 g/L trypsin (Yeason, China). Then the digest buffer was removed and the samples were cultured with Dulbecco's modified eagle medium (DMEM; Gibco, USA) containing 10% foetal bovine serum (FBS; Gibco, USA), followed by filtering with a 200-mesh copper mesh. The obtained cardiac fibroblasts were then cultivated in a complete medium (37°C, 5% CO_2_). For the CF model, cardiac fibroblasts were treated with 100 nM angiotensin II for 24 h to induce an in vitro myocardial fibrosis model.

### 2.3. Real-Time PCR

TRIzol agent (Thermo Fisher, USA)-isolated RNA from the treated myocardial tissue or cardiac fibroblasts was subjected to reverse transcription to obtain cDNA with the use of Reverse transcription kit (Takara, China). Real-time polymerase chain reaction (RT-PCR) was then carried out via a fluorescent quantitative PCR system (ABI, USA) to identify the expression of each mRNA in myocardial tissue or cardiac fibroblasts. The sequences of the genes and primers to be tested are listed in Table 1.

### 2.4. Western Blotting

The myocardial tissue or myocardial fibroblasts of each group were lysed with RIPA buffer to obtain total protein. The bicinchoninic acid (BCA) kit (Solarbio, China) was used to quantify the protein concentration of each sample. Then, 20 *μ*g protein extracted were separated by sodium dodecyl sulfate-polyacrylamide gel electrophoresis (SDS-PAGE), and transferred to a polyvinylidene fluoride (PVDF) membrane (Millipore, USA). After 1 hour of blocking in 5% skimmed milk, the PVDF membrane was incubated overnight at 4°C with primary antibodies GPX4 (1 : 1000, Abcam, UK), COX2 (1 : 1000, Abcam, UK), ACSL4 (1 : 10000, Abcam, UK), PTGS2 (1 : 1000, Abcam, UK), collagen I (1 : 1000, Abcam, UK), TGF-*β*1 (1 : 1000, Abcam, UK) and ACTIN (1 : 1000, Abcam, UK). Then came 1 hour of incubation with horseradish peroxidase conjugated secondary antibody at room temperature. Finally, the proteins were visualized using an enhanced chemiluminescent (ECL) kit (Yeason, China) and semiquantitative analysis was performed using the Tanon Imaging System (Tanon, China).

The article "MiR-375-3p Promotes Cardiac Fibrosis by Regulating the Ferroptosis Mediated by GPX4" was retracted in 2023. Reasons: signs of a paper mill; compromised peer review; unreliable results or conclusions.

### 2.5. Luciferase Assay

The binding of miR-375-3p to GPX4 mRNA was tested with the use of the Dual Luciferase Reporter Gene Assay Kit (Yeason, China). Then, the 3'UTR and mutation regions of GPX4 mRNA were cloned into the luciferase vector of pMIR-REPORT. MiR-375-3p and luciferase vector were coexpressed in cardiac fibroblasts. After that, 20 *μ*L cell lysate was added to the black microplate. Finally, 100 *μ*L firefly as well as renilla luciferase reaction solution were added to the plate to detect firefly and renilla luciferase activities.

### 2.6. Echocardiogram

Echocardiography was used to evaluate the cardiac structure and function of rats in each group. Four weeks after modeling, the rats were under isoflurane anesthesia to measure the left ventricular end-diastolic diameter (LVEDd), left ventricular ejection fraction (LVEF), left ventricular end-systolic diameter (LVESd), and left ventricular short axis shortening rate (LVFS) using a small animal color Doppler ultrasound system (BL-420S; Chengdu TaimengTechnology Co., Ltd.).

### 2.7. CCK8 Assay

The cardiac fibroblasts of each treatment group were seeded onto 96-well plates (10^4^ cells/well) for 24, 48 and 72 hours. After the addition of CCK-8 solution (10 *μ*L; Dojindo Laboratories, Japan) to each well, the cell viability at 450 nm was examined with a microplate reader. The testing of cell viability was performed at an interval of 24 hours.

### 2.8. Histological Staining

For hematoxylin-eosin (HE) staining, paraformaldehyde-fixed heart tissue was paraffin-embedded. With a paraffin microtome (Leica, Switzerland), the tissue block was cut into 2 *μ*m thick sections, which were then deparaffinized with xylene twice, rehydrated with ethanol gradient, and stained with hematoxylin (Beyotime Biotechnology, China) and eosin (Beyotime Biotechnology, China). Masson staining was performed according to the instructions provided by the reagent supplier (Solarbio, China). Specifically, after 10 minutes of dyeing with Weigert iron hematoxylin staining solution, the tissue sections were dyed with acid alcohol differentiation solution, Masson blue solution, and Ponceau magenta staining solution. After that, they were rinsed with weak acid and phosphomolybdic acid solutions, dyed with aniline blue staining solution for 2 minutes, and dehydrated with ethanol. All sections were blocked with neutral resin for microscopical observation.

The article "MiR-375-3p Promotes Cardiac Fibrosis by Regulating the Ferroptosis Mediated by GPX4" was retracted in 2023. Reasons: signs of a paper mill; compromised peer review; unreliable results or conclusions.

### 2.9. Antioxidant Content Determination

Myocardial tissue or myocardial fibroblasts were lysed by RIPA buffer to obtain a lysate. The levels of malondialdehyde (MDA) and superoxide dismutase (SOD) in myocardial tissue or myocardial fibroblast lysate were tested following the relevant instructions (Nanjing Jiancheng Biotechnology, China). The MDA content in the lysate at 532 nm and the SOD content at 450 nm were detected with a microplate reader.

## 3. Immunofluorescence

The treated cardiac fibroblasts were fixed with 4% paraformaldehyde for 15 minutes, rinsed with PBS, and permeabilized with 0.1% (v/v) Triton X-100 for 30 minutes at room temperature. Then the goat serum was dropped onto the cell slide and blocked at room temperature for 15 minutes. The slides were then added with anti-GPX4 antibody (1 : 100) or anti-ACSL4 antibody (1 : 100) for overnight incubation at 4°C. Following the addition of mGFP or mCheery labeled fluorescent secondary antibody, the slides were cultured at ambient temperature for 1 hour. DAPI was added dropwise for 5 minutes of cultivation, and the slides were sealed with antifluorescence quencher. The images were collected under a fluorescence microscope.

### 3.1. ROS Assay

ROS levels in cardiac fibroblasts were determined using ROS assay kits (Beyotime Biotechnology, China). The diluted DCFH-DA was added to the cultured fibroblasts. The cells were then washed with PBS 3 times to remove free DCFH-DA. The cardiac fibroblasts were then trypsinized and made into a cell suspension. The fluorescence intensity of DCFH-DA in the cell suspension was examined at excitation and emission wavelength of 500 and 525 nm, respectively.

### 3.2. Statistical Analysis

GraphPad software 7.0 was used for statistical analysis. The T-test was used for statistical comparison between two sets of samples. For statistical analysis of categorical data of three groups and above, one-way analysis of variance (ANOVA) was used. The significance level was *P* < 0.05 in this paper.

## 4. Results

### 4.1. MiR-375-3p Targets GPX4-Related Ferroptosis to Promote CF

We determined the expression level of miR-375-3p by RT-PCR in rat myocardial tissues of I/R group and sham group. The results showed that the expression of miR-375-3p was significantly upregulated in the I/R group compared with the sham group (Figure 1(a)). The expression of GPX4 was reduced, while the expression levels of COX2, ACSL4 and PTGS4 were increased in myocardial tissue of rats after IR injury (Figures 1(b) and 1(c)). This indicated that I/R injury induced myocardial tissue ferroptosis. I/R injury also upregulated the expression of collagen I and TGF-*β*1, indicating that CF was aggravated following I/R (Figures 1(b) and 1(c)). In the angiotensin II-induced CF model, miR-375-3p in cardiac fibroblasts after CF induction increased (Figure 1(d)) and the protein of GPX4 decreased (Figure 1(e) and 1(f)), versus the control group. The detection of ferroptosis and CF-related proteins showed that CF elevated the expression of COX2, ACSL4, PTGS2, collagen I and TGF-*β*1 (Figures 1(e) and 1(f)). In vitro, the proliferation rate of CF model cells was slower than that of normal fibroblasts (Figure 1(g)). The ROS assay revealed significantly increased ROS accumulation in CF model cells. Furthermore, we predicted the target genes of miR-375-3p and verified them through the luciferase reporter gene activity assay. The data revealed that miR-375-3p significantly down-regulated GPX4 mRNA reporter gene expression in cardiac fibroblasts but had no effect on 3'UTR mutant of GPX4 mRNA. This indicates that through directly targeting and down-regulating GPX4, miR-375-3p promotes the occurrence of CF by accelerating the ferroptosis of cardiomyocytes.

The article "MiR-375-3p Promotes Cardiac Fibrosis by Regulating the Ferroptosis Mediated by GPX4" was retracted in 2023. Reasons: signs of a paper mill; compromised peer review; unreliable results or conclusions.

### 4.2. Inhibition of MiR-375-3p and Ferroptosis Pathway Alleviates CF in an IR Model

We observed a significant reduction in miR-375-3p expression level and an increase of GPX4 expression level after treatment with Fer-1 and miR-375-3p inhibitor. We treated the I/R rat model with miR-375-3p inhibitor or ferroptosis inhibitor Fer-1. Imaging of the coronary arteries of rats and subsequent quantification of infarction showed that miR-375-3p inhibitor and Fer-1 significantly alleviated I/R-induced coronary infarction (Figure 2(a) and 2(b)). The results of Doppler echocardiography performed on the I/R rat model before and after treatment showed that miR-375-3p inhibitor and Fer-1 significantly reduced LVEF and LVFS, but increased LVIDs and LVIDd (Figures 2(c) and 2(d)). HE and MASSON staining of myocardial tissue showed that miR-375-3p inhibitor and Fer-1 significantly reduced myocardial fibrosis in rats (Figure 2(e)). Histological antioxidant assays showed that miR-375-3p antagomir and Fer-1 reduced I/R-induced MDA levels and increased SOD levels (Figure 2(f)). In the ferroptosis pathway, miR-375-3p antagomir and Fer-1 reduced I/R-induced iron levels and ROS levels (Figure 2(f)). In summary, miR-375-3p inhibitor and Fer-1 can alleviate I/R-induced CF.

The article "MiR-375-3p Promotes Cardiac Fibrosis by Regulating the Ferroptosis Mediated by GPX4" was retracted in 2023. Reasons: signs of a paper mill; compromised peer review; unreliable results or conclusions.

### 4.3. Inhibition of MiR-375-3p and Ferroptosis Pathway Improves Cellular Antioxidant Effect during Fibrosis in a Cardiac Fibroblast Model

Angiotensin II-induced cardiac fibroblasts were used to simulate fibrosis after MI, based on which the effect of Fer-1 and miR-375-3p inhibitor was evaluated. The results showed that both Fer-1 and miR-375-3p inhibitor promoted the viability of cardiac fibroblasts (Figure 3(a)). ELISA results showed that both Fer-1 and miR-375-3p inhibitor reduced the level of MDA and increased the level of SOD (Figure 3(b)). In the ferroptosis pathway, miR-375-3p inhibitor and Fer-1 reduced iron levels in the cardiac fibroblast model (Figure 3(b)). As a direct inducer of ferroptosis, intracellular ROS in cardiac fibroblasts was significantly reduced after miR-375-3p inhibitor or Fer-1 treatment (Figure 3(c)). It suggests that Fer-1 and miR-375-3p inhibitor promote the antioxidant capacity of the cardiac fibroblast model.

### 4.4. MiR-375-3p Inhibitor Relieves GPX4-Related Ferroptosis Process in a Cardiac Fibroblast Model

In angiotensin II-induced cardiac fibroblasts, we examined the changes in the GPX4-related ferroptosis process during the development of fibrosis. A significant reduction in miR-375-3p expression level and an increase in GPX4 expression level were observed after treatment with Fer-1 and miR-375-3p inhibitor. Among ferroptosis-related factors, miR-375-3p inhibitor and Fer-1 reduced mRNA levels of COX2, ACSL4 and PTGS2 (Figure 4(a)). Similarly, miR-375-3p inhibitor and Fer-1 elevated GPX4 protein, and lowered COX2, ACSL4 and PTGS2 protein expression (Figure 4(b)). Immunofluorescence results showed increased GPX4 protein in cardiac fibroblasts and decreased ACSL4 by miR-375-3p inhibitor and Fer-1 (Figure 4(c)). Therefore, miR-375-3p inhibitor and Fer-1 can reduce miR-375-3p expression and the ferroptosis process associated with GPX4.

### 4.5. MiR-375-3p Antagomir Alleviates GPX4-Related Ferroptosis in a Rat I/R Model

In the rat I/R model, the effects of miR-375-3p antagomir and Fer-1 on GPX4-related ferroptosis process were investigated. The results showed down-regulated miR-375-3p in the myocardial tissue of I/R rats and upregulated GPX4 mRNA after the intervention of miR-375-3p antagomir and Fer-1. Among the factors related to ferroptosis, miR-375-3p antagomir and Fer-1 reduced the mRNA levels of COX2, ACSL4 and PTGS2 (Figure 5(a)). Increased GPX4 protein expression and decreased COX2, ACSL4, and PTGS2 protein expression were also observed (Figure 5(b)). Immunofluorescence of rat myocardial tissue showed that miR-375-3p antagomir and Fer-1 increased the expression of GPX4 protein in myocardial tissue and decreased the expression of ACSL4 (Figure 5(c)). The results indicate that miR-375-3p antagomir and Fer-1 reduces the expression of miR-375-3p in myocardial tissue and the ferroptosis process associated with GPX4 in the I/R rat model.

The article "MiR-375-3p Promotes Cardiac Fibrosis by Regulating the Ferroptosis Mediated by GPX4" was retracted in 2023. Reasons: signs of a paper mill; compromised peer review; unreliable results or conclusions.

## 5. Discussion

Myocardial fibrosis is an important pathological change in various cardiovascular diseases. Many studies have shown that miRNAs are involved in myocardial fibroblast proliferation and collagen deposition in the progression of CF [23, 24]. For example, miR-125b is reported to enhance the proliferation of cardiac fibroblasts and the expression of Collagen I by targeting the expression of TP53 [25]. Transgenic mice expressing miR-328 specifically in the myocardium enhanced collagen deposition and induced CF by activating the TGF-*β*1 pathway [26]. Collagen production is one of the signs of myocardial fibrosis, and inhibiting the synthesis of collagen can also effectively reduce myocardial fibrosis [27]. It is shown that NLRP1 promoted the overproduction of collagen in neonatal cardiac fibroblasts and promoted myocardial fibrosis by directly targeting the TGF-*β*1/Smad signaling pathway [28]. In our study, miR-375-3p was observed to be highly expressed in I/R rat and CF cell models, and was closely related to severe myocardial fibrosis. In the CF model, we believe that elevated miR-375-3p expression was significantly associated with increased Collagen I expression. These studies and our data suggest that miR-375-3p can be a potential marker for CF treatment.

Ferroptosis is an important form of cardiomyocyte death. In some pathological conditions of the heart, excessive accumulation of iron ions, production of ROS, and pathological changes of membrane lipids are all important factors constituting ferroptosis [29]. Studies have revealed excessive ROS, lipid peroxidation and iron accumulation during cardiac ischemia and reperfusion [30, 31]. The ferroptosis inhibitor Fer-1 and iron chelator can effectively prevent ferroptosis-mediated heart damage [32]. In terms of mechanism, inhibition of glutamine metabolism can inhibit ferroptosis in the cardiac IR model, thereby alleviating cardiac injury [33]. In the formation of myocardial fibrosis, miR-351 targeted MLK3 to regulate the NF-*κ*B/NLRP3 signaling in myocardium and improved the cardiac function of mice with myocardial fibrosis [34]. Our research confirmed the regulatory role of miR-375-3p/GPX4 signaling in I/R rats and myocardial fibrosis transition, the mechanism of which is through the regulation of GPX4-mediated ferroptosis in cardiomyocytes. Ferroptosis intervention targeting the miR-375-3p/GPX4 signaling pathway provides a new approach for the prevention and treatment of heart diseases such as MI and fibrosis.

The article "MiR-375-3p Promotes Cardiac Fibrosis by Regulating the Ferroptosis Mediated by GPX4" was retracted in 2023. Reasons: signs of a paper mill; compromised peer review; unreliable results or conclusions.

The excessive deposition of ROS produced by oxidative stress leads to lipid peroxidation and DNA damage, which is the cause of severe pathological changes in the cardiovascular system. A large amount of evidence has found that ROS plays a key role in I/R injury and myocardial fibrosis [35–37]. GPX4, SOD and catalase can inhibit the toxicity of ROS [38]. In the process of redox scavenging ROS, GPX4 reduces the deposited ROS to the corresponding alcohol and water under the action of GSH [39]. The loss of GPX4 leads to mitochondrial dysfunction, which is manifested as decreased lipid oxidation capacity and increased ROS [40]. Therefore, GPX4 is a critical factor in mitochondrial metabolism disorders of cardiac cells. Doxorubicin (DOX) downregulation of GPX4 induces the formation of DOX-Fe2+ complexes in mitochondria, leading to excessive lipid peroxidation, which is directly related to myocardial fibrosis [41]. Our data showed that miR-375-3p-induced downregulation of GPX4 led to an increase in ROS and inhibited the oxidative scavenging effect of SOD. Therefore, miR-375-3p-mediated excessive oxidation may be the mechanism of CF development.

## 6. Conclusion

MiR-375-3p is an important factor inducing myocardial fibrosis after MI, which accelerates the ferroptosis of cardiomyocytes and promotes fibrosis by down-regulating GPX4. Meanwhile, this process can be reversed by miR-375-3p inhibitor or ferroptosis inhibitors. Therefore, the intervention of the miR-375-3p/GPX4 signaling pathway can alleviate IR-induced CF via reducing ferroptosis in cardiomyocytes, which provides potential approaches for clinical treatment of CF.

## Figures and Tables

**Figure 1:** MiR-375-3p directly targets GPX4 to promote ferroptosis and cardiac fibrosis. (a) RNA was extracted from the myocardial tissues of rats in the sham operation group (sham) and ischemia-reperfusion group (I/R), and the expression of miR-375-3p was detected by RT-PCR. (b) Western blotting was used to detect the expression of ferroptosis- and fibrosis-related proteins in the myocardial tissues of 3 cases of sham group and I/R group. The expression of each protein was quantified. (c) RT-PCR was used to detect the expression of genes related to ferroptosis and fibrosis. (d) RNA of normal cardiac fibroblasts (control) and cardiac fibroblasts induced by angiotensin II (CF model) were extracted, and the expression of miR-375-3p was detected by RT-PCR. (e) Western blotting was used to detect the expression of ferroptosis- and fibrosis-related proteins in control fibroblasts and CF models. The expression of each protein was quantified. (f) RT-PCR was used to detect the expression of ferroptosis- and fibrosis-related genes in control fibroblasts and CF model cells. (g) Control fibroblasts and CF model cells were cultured for 24 hours, and cell viability was assessed by CCK8. (h) The level of ROS in the control and CF model cells was measured. (i) Luciferase reporter gene activity was used to detect the binding of miR-375-3p to the 3'UTR region or mutant 3'UTR region of GPX4 mRNA. *Note.*^*∗*^*P* < 0.05, ^*∗∗*^*P* < 0.01 compared with the control group.

The article "MiR-375-3p Promotes Cardiac Fibrosis by Regulating the Ferroptosis Mediated by GPX4" was retracted in 2023. Reasons: signs of a paper mill; compromised peer review; unreliable results or conclusions.

**Figure 2:** MiR-375-3p inhibitor and ferrostatin-1 alleviate cardiac fibrosis in an I/R rat model. (a) The coronary artery stenosis of rats in the sham operation group (sham), I/R group, miRNA NC inhibitor treatment group, miR-375-3p inhibitor treatment group and Fer-1 treatment group was monitored by coronary artery imaging. (b) Quantitative analysis of the degree of coronary artery infarction in each group of rats. (c) Echocardiographic examination of rats in each treatment group. (d) Quantitative assessment of LVEF, LVFS, LVIDs and LVIDd of rats in each treatment group. (e) HE and Masson staining of myocardial tissue of rats in each treatment group. (f) Levels of MDA, SOD, iron ion and ROS in the myocardial tissue of rats in each treatment group. *Note.*^*∗*^*P* < 0.05 vs. sham, ^*∗∗*^*P* < 0.01 vs. sham, ^*##*^*P* < 0.01 vs. I/R and NC antagomir.

**Figure 3:** MiR-375-3p inhibitor and Ferrostatin-1 improve antioxidation during fibrosis of cardiac fibroblasts (a) Control fibroblasts, CF model cells, miRNA NC inhibitor treatment group, miR-375-3p inhibitor treatment group, and Fer-1 treatment group cells were cultured for 24–72 hours, and cell viability was assessed by CCK8. (b) Detection results of MDA, SOD, and iron contents in cells of each treatment group. (c) Determination and quantitative statistics of ROS content in cells of each treatment group. *Note.*^*∗*^*P* < 0.05 vs. control, ^*∗∗*^*P* < 0.01 vs. control, ^#^*P* < 0.05 vs. model and NC inhibitor, ^##^*P* < 0.01 vs. model and NC inhibitor.

**Figure 4:** MiR-375-3p inhibitor alleviates the GPX4-related ferroptosis process in a cardiac fibroblast model (a). RNA of control fibroblasts, CF model cells, miRNA NC inhibitor treatment group, miR-375-3p inhibitor treatment group and Fer-1 treatment group were extracted, and miR-375-3p and mRNA levels of GPX4, COX2, ACSL4 and PTGS2 were detected by RT-PCR. (b). Western blotting was used to detect the protein expression of GPX4, COX2, ACSL4 and PTGS2 in cells of each treatment group. (c). Immunofluorescence was used to detect the protein levels of GPX4 (red signal) and ACSL4 (green signal) in cells of each treatment group. DAPI was used to display the nucleus morphology. *Note.*^*∗*^*P* < 0.05 vs. control, ^*∗∗*^*P* < 0.01 vs. control, ^#^*P* < 0.01 vs. model and NC inhibitor, ^##^*P* < 0.01 model and NC inhibitor.

The article "MiR-375-3p Promotes Cardiac Fibrosis by Regulating the Ferroptosis Mediated by GPX4" was retracted in 2023. Reasons: signs of a paper mill; compromised peer review; unreliable results or conclusions.

**Figure 5:** MiR-375-3p antagomir alleviates the GPX4-related ferroptosis process in the I/R rat model. (a) RNA in the myocardial tissues of the sham operation group (sham), I/R group, miRNA NC inhibitor treatment group, miR-375-3p antagomir treatment group and Fer-1 treatment group was extracted, and miR-375-3p level and mRNA levels of GPX4, COX2, ACSL4 and PTGS2 was detected by RT-PCR. (b) Western blotting was used to detect the protein expression of GPX4, COX2, ACSL4 and PTGS2 in each treatment group. (c) Immunofluorescence was used to detect the protein levels of GPX4 (red) and ACSL4 (green) in the tissues of each treatment group. DAPI was used to display the nucleus morphology. *Note.*^*∗*^*P* < 0.05 vs. control, ^*∗∗*^*P* < 0.01 vs. control, ^#^*P* < 0.01 vs. model and NC inhibitor, ^##^*P* < 0.01 vs. model and NC inhibitor.

**Table 1:** Primers and sequences for RT-PCR.

Primer	Sequence
miR-375-3p	AAACAAGCTTGCCGTGCGCTCT
miR-U6- forward	CTCGCTTCGGCAGCACA
miR-U6- reverse	AACGCTTCACGAATTTGCGT
GPX4 forward	ACGCCAAAGTCCTAGGAAGC
GPX4 reverse	CTGCGAATTCGTGCATGGAG
COX2 forward	TGACTGTACCCGGACTGGAT
COX2 reverse	CATGGGAGTTGGGCAGTCAT
ACSL4 forward	TGAGCGCATACCTGGATTAGG
ACSL4 reverse	GCGCCAACTCTTCCAGTAGT
PTGS2 forward	CCGGACTGGATTCTACGGTG
PTGS2 reverse	ACTCTGTTGTGCTCCCGAAG
ACTIN forward	GGAGAAGATTTGGCACCACAC
ACTIN reverse	ACACAGCCTGGATGGCTACG

## Data Availability

All datasets generated for this study are included in the article.
